# Life Cycle Assessment of Construction and Demolition Waste from Railway Engineering Projects

**DOI:** 10.1155/2022/6145755

**Published:** 2022-04-28

**Authors:** Jianling Huang, Yang Yin, Lei Zheng, Sibo Zhang, Qingyun Zhao, Huihua Chen

**Affiliations:** ^1^School of Civil Engineering, Central South University, Changsha, China; ^2^School of Civil Engineering, Anhui Jianzhu University, Hefei, China

## Abstract

Railway engineering generates large amounts of construction and demolition waste (CDW). To quantify the amount of CDW generated from railway engineering projects throughout the whole life cycle, a process-based life cycle assessment model is proposed in this paper. The life-cycle CDW is divided into four parts: CDW from off-site transportation of construction materials (OSTCM), CDW from site operation wastage of construction materials (SOWCM), discard ballast from roadbeds, stationyard, bridges and tunnels (DB), and CDW from reparation and renewal of aging components (RRAC). Yun-Gui Railway is selected as a case study to validate the developed model, and an uncertainty analysis is conducted with Oracle Crystal Ball software. The results show that between 175 and 311 million tons of CDW is generated throughout the whole life cycle of Yun-Gui Railway. DB is the largest component of the life-cycle CDW from railway engineering projects. This indicates the negative environmental impacts of railway construction can be significantly mitigated by optimizing the location of ballast disposal sites and developing suitable landfill proposals. Also, the CDW generated by wastage of construction materials during off-site construction and site operation is important in waste management in railway engineering projects, in which rubble, sand, and cement have the high potential for waste reduction. Findings from this study can contribute to the knowledge body as well as the engineering practice in green railways.

## 1. Introduction

Construction and demolition waste (CDW) refers to the solid waste consisting of various surplus materials generated during the process of clearance, excavation, construction, refurbishment, and renovation [1, 2]. It is reported that approximately 10 billion tons of CDW is generated per year around the world [3], accounting for between 16 and 60% of landfilled waste worldwide [4, 5]. In Spain, Sáez et al. studied the CDW generation rate of new residential buildings in Spain. As shown in the study, 0.075 m^3^ of CDW is generated for every square meter of built surface of new residential construction, and waste coming from timber represented 31% of the total volume generated, followed by 16% of concrete and 13% of the mixture of concrete, tiles, and ceramic materials without hazardous materials [6]. In Malaysia, Mah et al. studied the CDW generation rate of different construction methods of high-rise buildings, and the study shows that the conventional construction method has a waste generation rate of 0.0988 t/m^2^, the mixed-construction method is 0.0329 t/m^2^, and demolition projects are 1.0428 t/m^2^ [7]. In Lebanon, daily construction waste generation ranges between 717 and 6353 tons in the Bekaa and Mount Lebanon governorates, respectively. The annual growth rate varied between 5.6 and 13%, with an average of 10-11% in most of the countries. As to demolition waste, a total of 810 tons is generated daily [8]. In Vietnam, construction waste generation rates of 79.3 kg/m^2^ and 1,030 kg/m^2^ were determined in small- and large-scale construction sites, respectively, while demolition waste generation rates at small and large demolition sites were 610 kg/m^2^ and 318 kg/m^2^ [9]. All these studies show that considering the amount of new floor space being built in countries around the world, the amount of construction waste generated is still huge and needs to be taken seriously. In China, with the rapid urbanization process and the growth of GDP, the total CDW increased rapidly. In 2018, the total CDW exceeded 1.8 billion tons and accounted for 30–40% of the total amount of urban waste. It is estimated that CDW of China will continue to increase at a rate of about 15% year by year, and by 2030, the total annual CDW is estimated to exceed 7 billion tons [10]. Up to now, many scholars have studied the generation of CDW. Hu et al. combined gray model with exponential smoothing method, took Chongqing metropolis as a case study, to estimate the annual output of CDW, and found that the main urban area of Chongqing will produce nearly 50 million tons of construction waste every year in the next 10 years, which is clearly beyond the capacity of the local CDW recycling plant [11]. Wang et al. used a unit building area method based on scenario analysis to predict CDW production in China Nanjing Jiangbei New Area for 2018 and 2019–2030. According to their research, Jiangbei New Area is expected to produce 5.92 million tons of construction waste and 44.87 million tons of demolition waste from 2019 to 2030 [12]. Wang et al. based on an empirical study, evaluated the waste generation rate of different types of waste at different construction stages by sorting and weighting the construction waste from 148 new-built residential construction sites on-site in China, and they found that the amount of inorganic nonmetallic waste with a generation rate of 16.59 kg/m^2^ was the highest among the five types of wastes (i.e., inorganic nonmetallic waste, organic waste, metallic waste, composite waste, and hazardous waste), while the waste generation rate for the underground construction stage, which was 27.57 kg/m^2^, was the highest among the three stages (i.e. underground stage, superstructure stage, and finishing stage) [13]. He et al. calculated the output of CDW in China from 2000 to 2016 by using CDW generation calculation method, and they proposed that China's construction waste generation will increase by 3% each year [14]. Tu et al. presented an estimation model of solid waste at construction site by means of decomposition-combined measurement, material tracking method, solid waste classification system, and mathematical analysis method. They estimated the amount of solid waste in different construction processes through using the model, and the calculation result show abandoned soil accounted for the largest proportion of the total solid waste, followed by concrete, masonry, wood, mortar, and metal [15]. All these studies show that Chinese annual CDW production presents an increasing trend year by year, and has not been paid enough attention to so far [16]. The continuous increase of CDW has caused serious adverse environmental and socioeconomic impacts. In conclusion, enhancing CDW management (CDWM) is vital for all economies in the world, both developing and developed countries.

China has the largest railway network in the world. By 2020, 37,929 kilometers of high-speed railways had been built in China, far more than in other countries, as shown in Table 1. Railway engineering has become a key part of infrastructure development under the background of the new era in China. By 2035, the length of China's railway network in operation is expected to reach about 200,000 kilometers, of which 70,000 kilometers will be high-speed railways (HSRs). This means China's railway engineering will maintain rapid development in the future. Compared with building projects, railway engineering projects have characteristics of trans-regional, large project scales, complex construction technologies, and difficult management. It is easy to generate a large amount of different CDW in the activities of earthwork, bridge construction, and tunnel excavation. Such a huge scale of China's railways must generate a lot of CDW, which decides CDW minimization through improved CDWM is the key to the sustainable development in railway engineering in China [17].

The reasonable methods to estimate the amount of generated CDW are the foundation of improving CDWM. Common methods for quantifying CDW include site survey (SS) method, generation rate calculation (GRC) method, lifetime analysis (LA) method, classification system accumulation (CSA) method, variables modeling (VM) method, and other particular methods [18]. SS method requires investigators to visit the construction or demolition sites for a realistic survey, and Lu et al. used this method to conduct on-site waste sorting and weighing in four ongoing construction projects in Shenzhen city of South China and obtained the generation rates and components of waste of Shenzhen [4]. GRC method is the most popular methodology, and the principle of it is to obtain the waste generation rate for a particular activity unit. Based on the method, Höglmeier calculated values of wood content of each of the 86 sample buildings and the amount of wood in the Bavarian building stock [19]. LA method is mainly implemented when quantifying demolition waste, and it is assumed that the amount of demolition waste must equal the mass of the constructed structure. Using this method, Cochran and Townsend predicted debris from demolition activities through the analysis of flows of materials during various activities in the lifetime of structures, based on the total amount, the average service lives, and the scrap rate during construction of construction materials consumed in the United States over time [20]. CSA method is developed based on GRC method, and the primary improvement is that CSA method involves a classification system, which provides a platform for quantifying different specified materials. Based on CSA method, Li and Zhang propose a web-based construction waste estimation system for building construction projects incorporating the concepts of work breakdown structure, material quantity takeoff, material classification, material conversion ratios, material wastage levels, and the mass balance principle [21]. VM method is using variables modeling to simulate the CDW generation, and using the method helps to understand the interrelationship among the variables. Katz and Baum developed a model that can predict the accumulation of construction waste by monitoring the amount and constituents of waste produced on 10 relatively large construction sites [22]. In many studies, more than one method might be applied comprehensively. Llatas, comprehensively using SV, GRC, and CSA methods, presented a model which allows technicians to estimate CDW during the design stage. The classification system of this model accords to the European Waste List (EWL), and the data was obtained from a four-floor 26 social housing building in Andalusia [23]. The above summary shows that the current research on the quantification of CDW is mainly focused on building projects, and the research focusing on railway engineering at the project level is still limited. There are three main reasons for this phenomenon: (1) Compared with the various forms of railway engineering, most building projects have little difference, which greatly facilitates the estimation of CDW. For example, using the GRC method and the waste generation rate of similar buildings, the amount of CDW of target buildings can be calculated quickly, while railway engineering cannot do this easy because of the lack of reliable data on CDW generation rates. (2) Building projects have fixed construction sites and relatively short construction period, which facilitates the research work related to CDW, including the quantification and management of CDW. (3) Generally, building projects are mostly located in urban areas, so for the consideration of urban environmental protection, the CDW management about them usually has higher requirements and needs more relevant studies also. In conclusion, the research on CDW quantitation about building projects has been relatively mature, while the research about railway engineering is still few. In order to accurately estimate railway engineering CDW, it is necessary to refer to the existing CDW quantification method to build a calculation model suitable for railway engineering CDW calculation.

Life cycle assessment (LCA) is a methodology to assess environmental impacts associated with all stages of a process or product throughout its life cycle from cradle to grave. According to standards defined by the International Organization for Standardization, a process-based LCA follows four steps: (1) goal and accounting scope definition, (2) inventory analysis, (3) environmental impact evaluation, and (4) results interpretation [24, 25]. For construction projects, the environmental impacts that are typically assessed in LCA research usually include greenhouse gas emissions, energy consumption [26], construction waste generation, etc. Based on these methodologies, many researchers conducted some studies on railways. Bortoli et al. proposed a set of 13 midpoint indicators to capture the diversity of the environmental damage of high-speed rail infrastructure by progressing a LCA model and a Life Cycle Inventories [27]. Banar and Ozdemir used LCA and Life Cycle Cost (LCC) methodologies to make an environmental and economic assessment of railway passenger transportation in the Turkish State Railway system, and the result shows that the impact of railways on the environment is caused mainly by infrastructure and operations [28]. Lin et al. used the hybrid economic input-output and LCA method to estimate the carbon footprints of different subsystems, different stages of production, and three calculation scopes of the Beijing-Shanghai high-speed railway line, and this study revealed nowadays China needs to make more measures to reduce the carbon footprints of HSRs [29]. Kaewunruen et al. used the LCA and LCC method to summarize the energy consumption, carbon emissions, and costs of the Beijing-Shanghai HSR, one of the most important railways in China, from the perspective of life cycle. It is concluded that the majority of the carbon emissions and energy consumption of the entire rail system comes from the construction stage [30]. Pons et al. evaluated the environmental impact of different railway track substructures including ballast, cast-in sleeper, and embedded track systems on the short-, medium-, and long-term by using the ReCiPe method to conduct a life cycle assessment of the railway infrastructure [31]. Akerman used a life cycle perspective to analyze the emission of the Europabanan, a high-speed rail track in Sweden, and found that the construction of new high-speed rail tracks will contribute to the reduction of carbon emissions [32]. Shinde et al. performed life cycle assessment for the Mumbai Suburban Railway by developing a comprehensive methodology for environmental evaluation of suburban railway projects in terms of energy consumption and relevant impact categories, and calculated the carbon emission of different stages and materials of railways [33]. Yue et al. based on the Chinese Core Life Cycle Database, conducted life cycle assessment of the Beijing-Shanghai high-speed railway line. The result shows that the vehicle operation stage dominates most impact of the emission of greenhouse gas which is mainly because the electricity mix in China heavily depends on coal-fired power generation [34]. Rungskunroch et al. analyzed five HSR networks from five countries by proposing a new critical framework, which is based on LCA and LCC models, capable of benchmarking the life cycle sustainability of HSR networks. The findings exhibit that key enabling policies related to ecofriendly rolling stock design, sustainable construction, and green energy grids play an important role in energy-saving of HSRs systems [35]. Jones et al. assessed the total life cycle environmental impact of the planned Portugal high-speed rail line from Lisbon to Porto by using the SimaPro Life Cycle Assessment software and found that the train operation process contributes the most to total environmental emissions [36]. In conclusion, most scholars currently use the LCA method to evaluate the energy consumption, carbon emission, and environmental impact of railway engineering, but few scholars estimate the CDW based on it. This is because railway engineering has a very long life cycle, including construction preparation stage, on-site construction stage, operation stage, and demolition stage, and railway engineering will produce a large number of CDW at each stage, which is different from construction engineering. So, compared with construction projects, it is much more difficult to estimate the CDW generated in the whole life cycle of railway engineering. However, only when the amount of CDW generated at each stage of the whole life cycle of railway engineering is calculated, can appropriate management measures to reduce CDW be formulated, which is crucial for China, which has a rapidly developing railway system. Based on this, the LCA method, which can analyze the generation of CDW from the perspective of the whole engineering, is used to estimate the amount of railway engineering CDW generation.

Based on literature review, this paper aims to develop a process-based LCA method for estimating the amount of CDW generated from railway engineering throughout its whole life cycle. This method bases on the material tracking method, and it calculates the CDW generated in each stage of railway project construction by analyzing the input, output, and flow of materials in the whole project. The idea of the method is that CDW comes from all kinds of materials that is put into the engineering; therefore, the amount of CDW generated at each stage can be calculated by analyzing the material inflow and the generation mode of CDW at each stage of railway construction. For example, in the construction preparation stage, the CDW is mainly generated by the off-site transportation of construction materials (OSTCM), so the total amount of CDW generated in this stage can be calculated by counting the total amount of all kinds of materials that need to be transported off-site and the loss rate of these materials in the transportation process. Compared with the traditional quantitative method, this method can obtain a more accurate calculation result. The reason is that railway projects are characterized by large quantities of engineering, many construction units, long construction period, etc. Traditional quantitative methods are difficult to accurately estimate the CDW generation. The estimation of CDW based on material tracking method can simplify the calculation process, avoid omissions in calculation, and investigate the type and amount of CDW generated at each stage of the railway project. A case in China is selected for demonstrating and validating the established model. The uncertainty analysis and sensitivity analysis are also conducted. Findings from this study can provide references for planning and construction of railway engineering especially in CDWM.

## 2. LCA Modeling for CDW Quantification in Railway Engineering

This paper develops a process-based quantitative LCA model for CDW generated from railway engineering projects based on the international standards ISO 14040 and ISO 14044 [24, 25]. It mainly consists of four interrelated steps: (1) goal and accounting scope definition; (2) inventory analysis; (3) environmental impact evaluation; (4) results interpretation.

### 2.1. Goal and Accounting Scope Definition

The first step in LCA research is to define the goal and accounting scope. It directly determines the extent of the study and is the most critical part of applying LCA. The goal of this paper is to estimate and quantify the amount of CDW generated from railway engineering projects throughout the whole life cycle. As shown in Figure 1, the life-cycle CDW of railway engineering projects includes three stages. Specifically, it includes the construction preparation stage, the on-site construction stage, and the operational stage. In the construction preparation stage, CDW is mainly caused by the OSTCM, such as the waste of rubble and sand in the transportation process. In addition, these losses are usually large and difficult to avoid. In on-site construction stage, CDW is mainly caused by the site operation wastage of construction materials (SOWCM) and the discard ballast from roadbeds, station yard, bridges, and tunnels (DB). SOWCM refers to the waste of materials caused by the use of them during construction, which is also difficult to avoid. DB refers to abandoned soil, discarded ballast, etc., resulted in roadbeds, station yard, bridges and tunnels construction. This discarded ballast is often huge and can easily be a waste of resources if not properly disposed of. In the operational stage, CDW mainly comes from reparation and renewal of aging components (RRAC). In railway engineering, it mainly refers to the maintenance and replacement of rails and their components. These are the important components of railway CDW, and there is no doubt that the demolition stage is also an important part of the whole life cycle of railway engineering. However, compared with building projects, the railway engineering projects generally do not have massive demolition after completion, but rather regular maintenance and replacement of rails, cables, and other components to ensure their long-term safe operation. In addition, when a passenger railway no longer meets operational requirements, it may be converted to freight rail for continued use. In other words, the life of a railway can last for hundreds of years sometimes. For these reasons, it is obvious that it is meaningless to calculate the amount of CDW produced in the demolition stage of railway engineering decades later and to formulate management measures. Thus, this study focuses on the CDW from the construction preparation stage, the on-site construction stage, and the operational stage, and the CDW from the demolition stage is not considered. The scope identification may also require continuous adjustment and refinement due to the repetitive nature of LCA analysis.

### 2.2. Inventory Analysis

The second step in LCA research is to compile an inventory of the system. This process emphasizes creating an inventory of the input and output data from the project. Collecting data and compiling a complete inventory based on the scope of the study as defined in the goal and accounting scope definition phase is the foundation of the LCA research. To quantify the amount of CDW generated throughout the whole life cycle of a railway engineering project, it is necessary to accurately interpret the design and construction plan, so as to obtain the precise statistics on the volume of work such as material consumption. This step is usually accomplished through methods such as on-site research and consulting engineering data. Also, it can be achieved by applying BIM, GIS, and other technical means.

### 2.3. Environmental Impact Evaluation

The third step is to analyze and evaluate the environmental impacts related to the life cycle of a product by using the compiled inventory. This process enables the transformation of the inventory data into specific impact types and indicators, thus providing a better understanding of the environmental impact on the life cycle of a product. Meanwhile, it is the basis of the results interpretation since it can provide the required information. According to the scope of the study and the complete inventory, the model for estimating the amount of CDW generated throughout the whole life cycle of a railway engineering project can be built.

This calculation model is based on material tracking method, and it calculates the amount of CDW by analyzing the material inflow and the generation mode of CDW at each stage of railway construction, as shown in Figure 2. The OSTCM can be calculated by multiplying the total amount of material to be transported by the damage rate of the material during transportation. The SOWCM is mainly caused by site operation of materials, so it can be calculated by multiplying the total amount of each material used in a railway engineering by the rate of loss of that material during use. DB is the discarded ballast from roadbeds, station yard, bridges, and tunnels, and it is determined by the total volume of excavation, fill taken of soil during the on-site construction. RRAC mainly comes from the replacement of waste materials in the operation stage of railway engineering, and it is mainly composed of unrecyclable parts of waste materials.

Based on the account scope determined above, the amount of the life-cycle CDW of a railway engineering project can be expressed as the sum of CDW generated in each stage, which is shown in

(1) $$\begin{array}{c} W=W_{T}+W_{C}+W_{S}+W_{R}, \end{array}$$

where *W* refers to the total amount of CDW generated throughout the life cycle of a railway engineering project; *W*_*T*_ are the amount of CDW from OSTCM in the construction preparation stage; *W*_*C*_ and *W*_*S*_, respectively, represent the amount of CDW from SOWCM and DB in the on-site construction stage; *W*_*R*_ refers to the amount of CDW from RRAC in the operational stage. The amount of CDW from each part can be calculated using Equations (2)–(5) according to the compiled inventory.

(2) $$\begin{array}{c} W_{T}=\sum_{i}^{n}W_{Ti}=\sum_{i}^{n}M_{i}*n_{Ti}, \end{array}$$

where *W*_*Ti*_ is the amount of CDW generated by the loss of the *i* − *th* construction material from OSTCM; *M*_*i*_ is the amount of the *i* − *th* construction material; *n*_*Ti*_ is waste rate due to OSTCM of the *i* − *th* construction material.

(3) $$\begin{array}{c} W_{C}=\sum_{i}^{n}W_{Ci}=\sum_{i}^{n}M_{i}*n_{Ci}, \end{array}$$

where *W*_*Ci*_ represents the amount of CDW generated by the loss of the *i* − *th* construction material from SOWCM; *M*_*i*_ is the amount of the *i* − *th* construction material; *n*_*Ci*_ is the waste rate due to SOWCM [37].

(4) $$\begin{array}{c} W_{S}=\left(V_{E}-V_{F}+V_{T}\right)*\rho_{S}, \end{array}$$

where *V*_*E*_ is the total volume of excavation during the on-site construction; *V*_*F*_ is total volume of fill during the on-site construction; *V*_*T*_ is the total volume of soil taken during the on-site construction; *ρ*_*S*_ is the average density of discard ballast. In this paper, the average density is set to be 2650 kg/m^3^.

(5) $$\begin{array}{c} W_{R}=\sum_{i}^{n}W_{Ri}=\sum_{i}^{n}\left(M_{i}-W_{Ti}-W_{Ci}-W_{Si}\right)*n_{i}*1-a_{i}, \end{array}$$

where *W*_*Ri*_ refers to the amount of CDW generated from RRAC; *M*_*i*_ is the amount of the *i* − *th* component; *n*_*i*_ is the number of replacements of the *i* − *th* component in the calculation period; *a*_*i*_ is the recovery rate of the *i* − *th* component [11]. In this paper, only steel recovery is considered and the recovery rate of steel is set to be 0.9.

### 2.4. Results Interpretation

The final step is to interpret the results. This step is based on the results of the inventory analysis and environmental impact evaluation to identify the major issues throughout the life cycle of a product and evaluate the results, whereby the conclusions, limitations, and recommendations are also formed. In this LCA research, the main materials and stages of CDW generated from railway engineering projects throughout the life cycle are identified. After identification, it can provide a reference for decision-making to enhance CDWM in railway engineering projects to achieve CDW reduction and resource utilization.

## 3. Case Study

### 3.1. Background Information

In this paper, Yun-Gui Railway is selected as a case study to demonstrate and validate the established quantitative model. This line is located in Yunnan and Guangxi provinces, from Kunming South Station to the east via Yuxi, Honghe, Wenshan, Baise, to Nanning Station, with a total length of 709.518 km. There are 259 new and reconstructed bridges, totaling 140.134 km and accounting for 19.75% of the total length of the line. Also, there are 184 new tunnels, totaling 430.772 km and accounting for 60.71% of the total length of the line.

### 3.2. Estimation Results

Based on the statistical analysis of the rail damage data of K807 + 000-K1110 + 000 section of Beijing-Guangzhou Railway from 2016 to 2018, Dai et al. estimated the rail fatigue life of 60 kg/m rails by establishing a three-dimensional solid finite element model. This study shows the number of rail damage increases nonlinearly with the increase of the total weight of the passed train and the fatigue life of 60 kg/m rails is about 1062 million tons to 1603 million tons [38]. According to the research results, the 60 kg/m rails are also used in the Yun-Gui Railway, 1300 million tons is taken as the average fatigue life of rails in this case study. Based on the estimated data of passenger and freight traffic of Yun-Gui Railway, the fatigue life of Yun-Gui railway rails was calculated, and the calculation shows the rails is expected to reach its fatigue life after 24 years of service [39]. In view of the corrosion of rails and the continuous increase of passenger and freight traffic, this study assumes 20 years as the average life of rails of Yun-Gui Railway. In addition, considering that the average life span of cables, metal strands, and other cable components used in railway engineering projects is about 15 to 20 years, the calculation period for LCA in this paper is taken as 20 years [40].

By collating the engineering information of Yun-Gui Railway, the inventory of each stage can be obtained, and the quantity of various materials and components is shown in Table 2. These provide the necessary database for LCA.

## 4. Discussions

The amount of CDW generated from Yun-Gui Railway throughout the life cycle is shown in Table 3. Approximately 243 million tons of CDW would be produced in the whole process, which is a huge amount and poses serious risks to the ecological environment along the line. Therefore, it is necessary to improve CDWM from the whole life cycle to achieve CDW reduction and resource utilization. In the whole life cycle, CDW generated from DB accounts for the highest proportion (up to 99%), which is the key to CDWM of railway engineering projects. It also proves the accuracy of the model calculation. In actual construction of railway projects, due to the existence of tunnel engineering, the generation of discard ballast is usually huge. However, the main components of the discarded ballast are soil and gravel, which are simple in composition and have relatively little negative impact on the environment. Hence, optimizing the location of ballast disposal sites and developing appropriate landfill schemes can decrease the pollution impacts on the environment. Other, the classified management and layered burial for ballast can facilitate the abandoned ballast backfilling project and the surrounding environment restoration project after the completion of the project, and reduce the impact of railway engineering on the surrounding environment. In addition to DB, a large amount of CDW would also be produced from OSTCM and SOWCM (1361500.68 tons and 1072825.11 tons). They are not as large as CDW generated from DB, but are also a significant amount. Reducing the loss and waste of construction materials by improving the construction material transportation process and construction sites is the key to achieving CDW reduction in railway engineering projects [41]. Compared to housing projects which generate a small percentage of CDW due to maintenance and renewal, the process of RRAC produces 313702.96 tons of CDW. This is because railways in the operation process will undertake much passenger and freight work, which can lead to wear and tear on rails and other components that need to be replaced regularly to ensure the safety of trains.

The proportion of CDW generated from different construction materials throughout the life cycle of Yun-Gui Railway is shown in Figure 3 (excluding discarded ballast). It can be learnt that rubble (37.5%), sand (29.7%), and cement (15.9%) contribute to the most proportion in the construction stage. This is because rubble, sand, and cement are consumed in great quantities during railway construction, and the losses are mainly caused by the transportation and use of the materials. This indicates that improving the transportation and use of these three materials can significantly reduce the production of CDW, which plays an important role in promoting CDW reduction in railway engineering projects. For example, much of the loss of rubble is caused by its transportation. In the actual construction process, the waste of rubble in the transportation process can be reduced by reducing the transport distance and choosing better transport vehicles. In the case of sand, improper transportation and storage mode can cause sand loss, so managers can reduce it through better storage methods and optimizing transportation timely. In addition, the percentage of rails is also high, accounting for 11.2%. The main reason is that the maintenance and renewal of rails during operation generates a great deal of waste [4]. As the core component supporting the train running, the state of rails is directly related to whether the trains can run normally. However, Yun-Gui Railway, as an essential channel in the southwest area of China, has a huge demand for passenger and freight transportation, which will accelerate the wear of rails. At present, there are few measures for rail recycling in China, and the rails that do not meet the requirements are mostly stacked in the warehouse [42]. This suggests that increasing the rail recycling can decrease unnecessary consumption. Other construction materials account for only 5.7% of the total. In general, the calculated results are consistent with the actual situation of railway CDW generation, which further proves the validity and accuracy of the calculation method.

In fact, the input parameters in this study such as material consumption are not exact constants. They are random variables due to the various types of errors that inevitably occur during the construction process. In order to further assess the possible range of CDW generation in the case project, an uncertainty analysis was carried out adopting Oracle Crystal Ball software, as shown in Figure 4. In this study, the weight of all kinds of materials flowing into the railway engineering and the discard ballast generated during construction is set as the input parameters due to they are the factors that can directly affect the amount of CDW. Also, it is assumed that the input parameters follow a standard normal distribution and the number of tests is set at 1 million. The results show that the amount of CDW generated approximately follows a normal distribution, with a variation range of 176506072.14 tons to 311143246.80 tons and a mean value of 243203018.36 tons. From this result, we can also find that the amount of CDW fluctuates greatly. It indicates that it is possible for us to take effective management measures to reduce the generation of CDW.

## 5. Conclusion

According to the process-based LCA theory, this study divides the sources of life-cycle CDW of railway engineering projects into four parts, namely, OSTCM, SOWCM, DB, and RRAC. This paper develops a LCA model to quantify the CDW generated from railway engineering. Yun-Gui Railway was selected to validate this model. The main conclusions drawn from this paper are as follows:

1. This study summarizes the existing CDW quantification methods and the research related to the LCA of railway engineering, and proposes a new railway engineering CDW calculation model based on material tracking method. Through the model, the amount of CDW generated at each stage can be calculated by analyzing the material inflow and the generation mode of CDW at each stage of railway construction.
2. A case study of Yun-Gui Railway shows that the entire line generates approximately 175 to 311 million tons of CDW, so it is urgent to strengthen the comprehensive management of CDW in railway engineering projects. In the whole life cycle of Yun-Gui Railway, the CDW generated from DB contributes the most proportion, which is considerably higher than the CDW generated from other phases. This indicates that optimizing the location of ballast disposal sites and developing appropriate landfill proposals can significantly mitigate the pollution caused by railway construction. The CDW generated from, OSTCM, DB, and RRAC account for a similar proportion. Therefore, it is meaningful to reduce the generation of CDW and achieve the goal of green railway construction by studying the generation mode and composition of CDW in each stage and formulating targeted recycling plan.
3. From the perspective of the amount of CDW generated by various construction materials throughout the life cycle of Yun-Gui Railway, rubble (37.5%), sand (29.7%), and cement (15.9%) are the most important sources of CDW. This is followed by tails, which account for 11.2% and are mainly generated for the maintenance and renewal of rails during the operational period. Other construction materials contribute a small amount, totaling only 5.7% of the total.

Although this paper has made some achievements in the calculation of railway CDW, there are still some shortcomings, as follows:

1. The calculation model proposed in the paper calculates the CDW generation mainly by multiplying the amount of material by the rate of material consumption. Therefore, for the model, an accurate and reliable CDW generation rate is crucial. The lack of CDW generation rate will lead to the failure of this calculation model, while it is difficult to get an accurate waste generation rate most of the time.
2. The definition of accounting scope in this study is not necessarily accurate. In the actual use of the calculation model, the accounting scope needs to be adjusted according to the characteristics of various railway engineering and the generation mode of CDW, so as to ensure the accuracy of the calculation of the total amount of CDW.
3. The results did not reflect the spatial and temporal distribution of railway CDW, although it is important for the formulation of waste management policies also.

In conclusion, the LCA model and BIM or GIS technology can be combined to explore the spatial and temporal distribution of CDW generation throughout the life cycle of railway engineering projects in the future.

## Figures and Tables

**Figure 1:** The life-cycle CDW of railway engineering projects.

**Figure 2:** The life-cycle material flow of railway engineering projects.

**Figure 3:** Proportion of life-cycle CDW generated from various construction materials.

**Figure 4:** The possible range of CDW generated from Yun-Gui railway (unit: tons).

**Table 1:** Length of high-speed lines of the major economies by 2020 (unit: km).

Country	Length
China	37929
France	10368
Japan	5236
Germany	2670
Korea	887
United States	735

Note: data are from UIC (an International Union of Railways, https://uic.org).

**Table 2:** Construction material consumption of Yun-Gui railway (unit: tons).

Material	Consumption	Material	Consumption
Cement	10932704	Steel moulding plate	17011
Explosive	36925	Steel braces	3410
Reinforced concrete pole	4793	Steel	1217268
Rubble	26734649	Cable	413
Sand	16341537	Steel stranded wire	25264
Lime	206672	Aluminum conductor steel reinforced	2086
Fly ash	1386389	Rail	287306
Ballast	1905540	Reinforced concrete sleeper	23443

**Table 3:** CDW generated in different life cycle stages from Yun-Gui railway (unit: tons).

CDW generation stage	Amount
OSTCM	1361501.68
SOWCM	240431320.00
DB	1072825.11
RRAC	313702.96

## Data Availability

All used data have been included in the manuscript.
